RETRACTED

# Analysis of Nostalgia Emotional Experience, Rural Tourism Environment Cognition, and Consumption Willingness Based on Big Data Technology

**DOI:** 10.1155/2022/2271650

**Published:** 2022-10-05

**Authors:** Wei Cao, Fanhui Meng

**Affiliations:** Chuzhou University, Chuzhou 239000, China

## Abstract

As the primary research vehicle, rural tourism is used in this paper to examine urban visitors' “homesickness.” This research explores the effects of homesickness on tourists' perceptions of travel destinations and consumption intentions through qualitative analysis, logistic empirical analysis, and questionnaire survey. This work also explores the behavioral traits of customers' purchase intentions from the perspective of a “big data” environment, and it constructs the relevant consumption behavior model for rural visitors in accordance with those behavioral traits. Through questionnaire design and investigation, this paper makes statistical analysis on tourists' basic information, expected value, and actual experience and explores the related factors that affect their consumption behavior, so as to understand the consumption behavior law of tourists in rural tourism consumption. The research shows that the MSE (mean squared error) of this algorithm is about 4.16, and the RMSE (root mean square error) of this algorithm is about 0.508. Finally, combining the influence of tourists' consumption behavior, this paper tries to put forward some countermeasures and suggestions on rural tourism. This paper aims to study the development and planning of rural tourist destinations, and provide corresponding basis for the destination selection of tourists with homesickness.

## 1. Introduction

Rural tourism with the theme of returning to rural natural scenery was created as a result of the economy's quick expansion, the level of urbanization's continual improvement, and the thorough development of tourism. Rural tourism is growing and developing as a result of tourism reaching a particular level of development and the need for product diversification in the industry. It satisfies urban dwellers' needs to reenter nature and relieve the intense pressure of daily life and work [1]. The position and role of tourism in relieving people's living pressure, improving people's living standard, stimulating domestic demand, and promoting residents' consumption are becoming increasingly prominent. The development of rural tourism can help to increase the employment rate, further increase farmers' income, optimize the local industrial structure, and promote the integration of urban and rural areas [2]. As the urban space is squeezed, more and more urban residents tend to travel to the countryside for holidays. However, nowadays, the decline and ruin of rural areas, the pressure and noise of cities, and the intensification of urban-rural contradictions have triggered people's deep reflection on rural governance. In this round of anti-ideological trend, the subject of “homesickness” has shifted from the cultural perspective to the public perspective [3]. With the emergence of big data, the technology in the world has changed greatly, and people's way of life and cognitive thinking in the world have had a great impact. The application value of big data lies not in the huge amount of data, but in how to utilize and mine these data, analyze the situation of tourism consumers, timely assess the impact of homesickness emotional experience on rural tourist destinations' cognition and consumption intention, and discover the practical significance behind tourism data [4]. The study of consumer behavior will be greatly impacted by the use of big data's technical tools given its rapid development [5]. Therefore, it is important from a practical standpoint to examine the cognition and consumption intention of homesickness emotional experience to rural tourist locations based on big data technology.

RETRACTED

Nowadays, the consumption patterns of consumers have undergone earth-shaking changes, while the rural tourism market is still in the primary development stage, and all aspects are not yet mature and perfect. On this basis, by studying consumer behavior and fully grasping the behavior rules of the tourist market, it is more conducive to the targeted development of rural tourism projects and provides feasible strategies for the development and development of rural tourism [6]. The real needs of consumers are hidden, complex, changeable, and environment-dependent. It is difficult for enterprises to obtain the real needs of users by using traditional, static, and structured data. “Big data” may give enterprises real consumer demand. According to the different perception of tourism information value, targeted marketing can improve the efficiency of marketing management and create more value with limited marketing resources [7]. There are many factors that affect tourism consumption, and generally speaking, they can be divided into two categories: (1) the factors of tourist destination and (2) the factors of tourists themselves. Among these factors, the main influencing factors on rural tourists' tourism consumption are destination charm, hardware factors, products and services, tourism resources, support systems, etc. from the awakening of rural consumers' tourism awareness to making tourism decisions and forming tourism experience and evaluation. In the whole process of tourism consumption, the psychological factors that affect the behavior of rural tourism consumers can be divided into two categories: (1) internal psychological factors, including perception, learning, personality, motivation, and attitude, and (2) social environmental factors, including culture, social class, family, and related groups. In order to improve the development level of rural tourism, we should pay attention to the needs of tourists and conduct in-depth research on their needs [8]. Only in this way can we provide the world's rural tourism industry exceptional solutions while eschewing irrational development practices and excessive development strategies. This article examines the influence of homesickness emotional experience on the cognition and consumption intention of rural tourist locations using big data technologies. The following are the innovations of this paper:

1. The impact of homesickness on tourist destination cognition and consumption intention is examined in this research by qualitative analysis, logistic empirical analysis, and questionnaire survey. In an effort to measure tourist loyalty comprehensively, it is planned to use both the positive intentions of returning, recommending, etc. and the negative intentions of looking for alternatives. It is more in line with tourists' objective psychological activities to study the correlation between each dimension under the subdivision dimension
2. This research examines the behavior traits of consumers' purchase intentions from the perspective of a “big data” environment, and as a result, it constructs the appropriate consumption behavior model of rural visitors. In addition to the impact of tourists' spending habits, this study also makes some recommendations and countermeasures for rural tourism

RETRACTED

## 2. Related Work

Loureiro thinks that the most fundamental reason for urban people to travel to the countryside on a large scale is their inner “local complex” [9], besides their yearning for tourism. Long et al. verified the influence of adjustment orientation and communication strategies on tourists' perceived value and purchase intention through two experiments according to the adjustment matching theory [10]. Iorio and Corsale pointed out that rural tourism is a phenomenon of tourism activities, which attracts the typical rural landscape resources and can meet the needs of tourists for seeking differences, knowledge, and roots [11]. It includes tourists' rural tourism activities, and the rural tourism landscape development and design activities carried out on this basis. Chen et al. found in the basic characteristic variables of the investigators that gender is negatively weakly correlated, age is positively weakly correlated, education level is strongly correlated, and travel form and choice mode are positively correlated [12]. Smith et al. think that in rural tourism, the essence of tourists' concern is rural culture, and the essence of rural areas' concern should be the inheritance and protection of rural culture [13]. Ahuja and Cooper improved the choice-based model, added emotional components on the basis of attribute evaluation, and measured consumers' willingness to buy products, which achieved good results [14]. According to Andres et al., rural communities are the foundation of rural tourism. Take into account the rural natural ecological environment, settlement patterns, economic patterns, and cultural patterns as tourism resources; consider the living conditions and way of life as an experience; farming is a type of ecotourism that is distinct from the local rural communities' residents and is geared toward the market [15]. With the emergence of some phenomena in rural tourism, such as the tension between people and land and the destruction of rural images, more scholars began to call for a return to the essence of rural tourism. Cruz et al. found that rural tourism was seriously damaged, and they regarded the cognition and protection of rural tourism as the essence of rural tourism [16]. From the viewpoint of tourists' consumption patterns, Muresan et al. sought to identify the distinctive rural tourism mode before proposing workable development strategies to support the long-term growth of rural tourism [17]. Based on information from web searches, Caruana et al. projected the tourist flow [18]. Additionally, the technique of substituting tourist hotspots in other areas is used to forecast the tourist flow in a certain site in order to assess the durability of the created model. According to Funk and colleagues, rural tourism alienates people from the land and prevents them from expressing their sentiments for it. The core of rural tourism is the restoration and regeneration of the current local-human structure [19]. From a sociological standpoint, He et al. incorporated theories and methodologies from economics, psychology, geography, and other fields to make scientific applications and selections [20]. The behavior model of rural tourists is also built in accordance with the peculiarities of their consumption patterns.

Although many academics have started to look at the issue from the standpoint of travellers' desires, the majority of them simply consider psychological motivation as a component of the “push” in the research of rural tourism motivation. The majority of research do not thoroughly examine how psychological and emotional factors influence the entire tourism consumption process. Beginning with the “homesickness” of urban visitors, this essay uses rural tourism as its primary study vehicle. The impact of homesickness on tourist destination cognition and consumption intention is examined in this research by qualitative analysis, logistic empirical analysis, and questionnaire survey. In addition, this study explores the behavior traits of consumers' purchasing intentions from the perspective of the “big data” environment and develops the corresponding sustainable development of rural ecotourism.

RETRACTED

## 3. Methodology

### 3.1. The Impact of Homesickness Emotional Experience on the Cognition and Consumption Willingness of Rural Tourist Destinations

At present, tourism plays a very important role in social and economic development. As a comprehensive modern service industry, tourism has become a very important force in the development of national economy. At the same time, with the advent of the Internet-based media era, people's public speech space is further expanded, and homesickness connects urbanites with rural people. In rural tourism, we found the unique feelings of tourists for the countryside. Rural tourism includes all aspects of tourism, that is, natural, social, and historical dimensions. This means that consumers' perception of rural areas, consumption in rural areas, and all kinds of tourism activities carried out by using rural space are called rural tourism according to their needs and demands. Tourism behavior comes from tourists' tourism motivation, which is the driving force of tourism behavior. Motivation comes from a certain need of people. It is the existence of unsatisfied desire or need that inspires the motivation to satisfy this desire, so the motivation of tourism is related to the level of people's needs. Tourists' perception of information value is closely related to tourism demand. Tourism information value is defined as tourists' evaluation of the importance of tourism information at the value level. It includes functional value and experiential value. Consumption runs through the whole tourism activities. In order to achieve the purpose of tourism, tourists must get reception services such as food, accommodation, transportation, shopping, and entertainment. Rural tourists' consumption behavior is a kind of behavior that is greatly influenced by internal and external factors. When rural tourists have consumption behavior, the “stimulus-response” theory effectively explains the potential impact perceived by tourists. Tourism decision-making process is the same as most other types of decision-making processes of consumers, and decision-makers often need to go through several psychological steps. The decision-making process mode is shown in Figure 1.

RETRACTED

In literary works and public life, homesickness is rich in content, but its specific elements are stable. In this paper, it can be roughly divided into three parts: hometown geography, cultural history, and ecological environment. From the perspective of the course of life, homesickness is often the patent of adults. The ultimate goal of tourists' travel is to get physical and mental enjoyment. Whether it is sightseeing, cultural tourism, vacation and leisure tourism, or ecotourism, the most fundamental pursuit of tourists is to relax their spirits, adjust their mood, increase their knowledge, and get enjoyment that is hard to get at home. Rural tourism products are the main objects for tourists to gain tourism experience. The main contents are sharing rural culture and rural life with local villagers in rural atmosphere, as well as rural reception and holiday services. Secondly, it is products provided by local people who are directly or indirectly engaged in tourism. Rural tourists buy a special service product, and the production and consumption of tourism products happen at the same time in different places, so tourists need a complicated evaluation process before purchasing. At the same time, tourism consumption is a kind of nonrecurring high-level consumption, and tourists often have to make careful choices. The length of a tourist's journey is determined by certain objective conditions. The most important conditions are time, expense, and discomfort of the journey. The research on tourism consumption behavior can be carried out from many angles, and there are two most representative research models: (1) the “need-motivation-behavior” model represented by Gilbert and (2) the “stimulus-response” model represented by Middleton. Although the above two models have different starting points and focuses, they blend with each other, and the factors that affect tourism consumption behavior are basically the same. The theory of consumption motivation points out that motivation comes from the stimulation of the human brain by the objective world. Consumers' motivation urges them to produce consumption behaviors, and different opportunities lead to different consumption behaviors. Therefore, tourists' emotion will affect their choice of tourism destination, and whether their emotional needs can be met or not will affect their attitude towards destination products and services. Nowadays, tourism activities, whether in the content or the purpose of tourism, are very comprehensive, so tourism consumption behavior also presents diversity, for example, sightseeing, entertainment, cultural tourism, nature tourism, business tourism, visiting relatives and friends, and health tourism. Consumer's purchase decision-making process refers to a series of processes during the selection, purchase, and experience of tourist products or services. The travel preparation stage before consumption refers to some choices that tourists need to make before arriving at the destination of rural tourism, that is, the consumption behavior in the preparation stage, including travel modes, cognitive channels, and peers. According to the actual situation, both travel expenses and travel discomfort are obtained after consumption, and tourists cannot grasp the specific information of these two aspects when making travel decisions. Therefore, in actual decision-making, the maximum distance of tourism should be the tangent point of tourists' time constraint line, consumption possibility line, and tourism indifference curve.  Figure 2 shows the best tourist distance.

RETRACTED

Tourists' “homesickness” will affect their expectations of rural tourism. In the process of tourism, tourists compare their perceptions with their expectations and get satisfaction evaluation results, which become an important reference for their willingness to revisit. The types of rural tourism products are different from region to region, from different forms of agricultural production, and from the distribution of ethnic groups. Different regions, climatic conditions, and topography are different, so there are different natural landscapes and agricultural production forms. Therefore, the types of products supplied by rural tourism are various. Tourists' perception, that is, tourism perception, refers to the overall reaction of tourism stimulus directly acting on sensory organs in human brain. Perception has the characteristics of selectivity, comprehension, integrity, and constancy, which is also the reason why tourists have different perceptions of the same type of tourism products. Although different types of tourists have different demand characteristics in terms of the length of travel time, the sensitivity of travel prices, and the choice of travel destinations, as the main body of travel activities, their travel consumption behaviors have some commonalities. Human behavior is the crystallization of personal characteristics and environmental effects. Tourism is also a kind of consumption behavior, and the travel experience of rural tourists also conforms to the theory of cognition-emotion-behavior will. Before choosing a rural tourism destination and making a travel decision, tourists usually use the Internet, relatives and friends, travel agencies, and other channels to make a preliminary cognition by using mobile phone information about rural tourism destinations. Personal psychological and physiological factors will have a certain impact on people's behavior. At the same time, people's psychological and physiological factors will have a certain impact on their cognition and evaluation of the tourism environment and their decision-making criteria. In the tourism consumption activities, tourism consumers with different temperament types, such as manners, reaction speed, nervous state, and a series of behaviors that show their temperament characteristics in different degrees, will directly affect their purchasing behavior and have a profound impact. In the rural tour stage, young people and old people will have exciting, novel, and challenging activities, respectively; a safe and quiet living environment is the core pursuit goal.

RETRACTED

### 3.2. Analysis of Consumers' Purchase Intention in Big Data Environment

People use the term “big data” to describe and categorize the vast amounts of data produced in the information age as well as to refer to associated technological advancements. Big data describes the enormous volume of data involved, which cannot be quickly collected, handled, processed, and categorized into information that can be understood by humans. Big data considerably improves event predictability due to its robust data analysis capabilities, which draws significant interest from all spheres of society. The behavior law of big data concealing is being raised out of the water as a result of the widespread use of big data. Big data is complicated and changing and contains a number of different data kinds because its primary data source is information that has been left over from the Internet. Data can take many different forms, including unstructured data like audio, video, photos, and geographic locations, as well as structured data like tables, semistructured data like web pages, and both, and create a “multisource heterogeneous” data type with unstructured as its main component. Big data's fundamental properties are typically thought to include six components as follows: intricacy, complexity, kind, speed, variability, and genuineness. Big data analysis allows for the segmentation of consumer behavior and the creation of customized marketing campaigns and services for each consumer group. Therefore, it is crucial for marketers from all backgrounds to learn the art of mining big data for its marketing potential. This article examines the effects of homesickness emotional experience on cognition and consumption willingness of rural tourism locations using big data technology.

RETRACTED

The construction of consumer behavior model aims at simplifying the relationship among all influencing factors of consumer behavior. In fact, the ultimate goal of the model is to describe consumer behavior and control its behavior pattern. The occurrence of tourism and activities should be based on the spatial movement of the actors. In fact, the process of tourists' travel is a process of constantly adjusting their own conditions to adapt to the natural and cultural environment in different places. To construct an analysis model of homesickness emotional experience's cognition and consumption intention of rural tourist destinations, it is necessary to create a corresponding structural model. The model needs to meet the following conditions: (1) It aims at the behavior characteristics of rural tourism consumers. (2) It starts from the consumption patterns of rural tourists. (3) Consider the dynamics of rural tourists' consumption decisions. (4) The model is superior to the previous models and can be verified in practice. Homesickness emotion is essentially the emotional characteristics of tourists when they face the countryside, and it is also in line with the general characteristics of tourism emotion. The design of homesickness scale for tourists in this paper is shown in Table 1.

According to Fishbein model, consumer attitudes about this particular object throughout the process are mostly determined by how strongly customers believe that various characteristics of goods or brands will perform as promised. The following formula specifically describes the Fishbein model:

(1) $$\begin{array}{c} A_{0}=\overset{N}{\underset{i=1}{\sum }}b_{i}e_{i}. \end{array}$$

Among them, *A*_0_ is the attitude of consumers towards a specific object; *b*_*i*_ is the strength of consumer's belief in the attribute *i* of the object; *e*_*i*_ is the evaluation of attribute *i*; *N* is the number of significant beliefs related to this object. Support degree is the probability that a certain set (*X*, *Y*) appears in the total set *I* shown as

(2) $$\begin{array}{c} \text{support}\left(X⟶Y\right)=\frac{P\left(X,Y\right)}{P\left(I\right)}=\frac{P\left(X\cup Y\right)}{P\left(I\right)}. \end{array}$$

Confidence indicates the probability of deducing *Y* according to association rules under the condition of *X* event. The formula is as follows:

(3) $$\begin{array}{c} \text{confidence}\left(X⟶Y\right)=P\left(Y\left|X\right.\right)=\frac{P\left(X,Y\right)}{P\left(X\right)}=\frac{P\left(X\cup Y\right)}{P\left(X\right)}. \end{array}$$

The degree of promotion indicates the ratio of the probability of containing *Y* under the condition of containing *X* to the probability of containing *Y* without *X*. The formula is as follows:

(4) $$\begin{array}{c} \text{lift}\left(X⟶Y\right)=\frac{P\left(Y\left|X\right.\right)}{P\left(Y\right)}. \end{array}$$

Let the benchmark index sequence be

(5) $$\begin{array}{c} y=\left(y_{1},y_{2}\cdots y_{n}\right). \end{array}$$

For any sequence satisfying *p*_*i*_ > 0, ∑*p*_*i*_ = 1, *p* can be used as the probability distribution sequence of a random variable. Therefore, it is necessary to standardize the benchmark index sequence and record the transformed sequence as *p*, namely

(6) $$\begin{array}{c} p_{t}=\frac{y_{t}}{\sum_{t=1}^{n}y},t=1,2\cdots n. \end{array}$$

The formula for calculating the amount of K-L information can be expressed as

(7) $$\begin{array}{c} I\left(p,q\right)=k_{1}=\overset{n}{\underset{i=1}{\sum }}p_{i}\ln\frac{p_{i}}{q_{i}},l=0,\pm 1,\pm 2\cdots \pm L. \end{array}$$

When the benchmark index sequence is consistent with the alternative index sequence, the information amount of K-L is zero; The closer an index is to the benchmark index, the closer the information content of K-L is to zero. Suppose the research object includes *n* samples and *p* variables (*n* > *p*), which are expressed as vectors:

(8) $$\begin{array}{c} X={\left(X_{1,}X_{2},\cdots ,X_{p}\right)}_{n\times p}. \end{array}$$

Linear transformation of *X* to form a new comprehensive index vector *Y*:

(9) $$\begin{array}{c} \left\{\begin{array}{c} Y_{1}=u_{11}X_{1}+u_{12}X_{2}+\cdots +u_{1p}X_{p},\\ Y_{2}=u_{21}X_{1}+u_{22}X_{2}+\cdots +u_{2p}X_{p},\\ \cdots \\ Y_{p}=u_{p1}X_{1}+u_{p2}X_{2}+\cdots +u_{pp}X_{p}. \end{array}\right. \end{array}$$

Among them, *u*_*k*1_^2^ + *u*_*k*2_^2^ + ⋯*u*_*kp*_^2^ = 1, *k* = 1, 2, ⋯, *p*.

RETRACTED

Because the original variables are linearly transformed as shown in formula (9), the characteristics of *p* comprehensive indicators obtained are not the same.

The theory of tourists' behavior pattern holds that tourists' completion of travel activities is mainly influenced by external and internal factors. The external factors include marketing factors and incentive factors, while the internal factors include tourists' characteristics and decision-making process. External stimuli and internal factors determine the outcome. Cluster analysis [21] is mainly based on the similarity of variables and objectively classifies the similarities into one class, which can make the same class have high homogeneity. In this paper, tourists' motivation is explored into a few factors, then the dimensions of tourists' motivation are established according to the factors, and then different types of tourists' motivation are distinguished by *K*-means cluster analysis. According to the origin of consumer behavior, this paper holds that the core part of consumer behavior research should cover the transition process from decision-making to the origin of consumer behavior, not only the characteristics of buyers and the decision-making process. The return of tourists from tourist destination to tourist residence means the end of this tourism activity, but the role played by this stage cannot be ignored. Tourists will recall and evaluate this tourism activity for a long time after returning to their place of residence [22]. If tourists are very satisfied with this trip, they will tend to buy this product and service next time. If tourists are dissatisfied, they tend not to buy the products and services.

RETRACTED

## 4. Result Analysis and Discussion

Tourism has obvious seasonal fluctuation. In order to enhance the representativeness of the survey population, this paper chooses to conduct market survey in the peak season of the research object. During the peak season, the probability of population types in various markets is high, and the sampling is convenient and scientific. The design of the scale is mainly based on summarizing and sorting out the measurement dimensions and questions involved in previous studies, which is the basis of designing the questionnaire in this paper. At the same time, according to the needs of this study, combined with the specific context of tourists' travel, the questions are modified to obtain the measurement scale used in this research. The basic information of tourists is an important part of the questionnaire, which lays a good foundation for in-depth research by mastering and understanding the source, sex, age, occupation, monthly income, and education level of the respondents. Descriptive statistical analysis was carried out by using SPSS17.0 software. See Table 2 for the specific sample situation.

That is, when the same object is measured again using the same method, reliability refers to the consistency of the data produced. An efficient analysis technique to gauge the consistency and stability of a thorough evaluation system is the reliability test. The dependability coefficient of Cronbach is the one that is currently most frequently utilized.  Table 3 displays the outcomes of the data reliability test used in this study.

Without screening, it is challenging to ensure the data's impartiality and integrity in the face of a vast volume of data; analysis and integration of data would invariably lose their value due to flaws. As a result, the data in this work are preprocessed before being divided into training, verification, and test sets. Raw data, data after data cleaning, and data after data expansion make up the training set. The algorithm is first tested using MSE and RMSE, with the following formula:

(10) $$\begin{array}{c} \text{MSE}=\frac{1}{n}\overset{n}{\underset{k=1}{\sum }}{\left(y_{k}-y\prime_{k}\right)}^{2},\\ \text{RMSE}=\sqrt{\frac{1}{n}\overset{n}{\underset{k=1}{\sum }}{\left(\left|y_{k}-y\prime_{k}\right|\right)}^{2}}. \end{array}$$

Among them, *y*_*k*_ is the actual value, and *y*′_*k*_ is the output value. The MSE results of different algorithms are shown in Figure 3. RMSE results of different algorithms are shown in Figure 4.

RETRACTED

It can be seen that the error of this algorithm is small. Then, the accuracy of this algorithm is tested, and the results are shown in Figure 5.

The core competitiveness of rural tourism destination comes from tourists' good perception of its value when traveling in this place, and tourists mainly perceive it from six aspects, namely: management and service, facilities, landscape, project, society, spirit, and cost.  Table 4 is descriptive statistics of rural tourists' attribute perception and emotional perception.

The empirical analysis is carried out on all samples. In order to verify the robustness of the relationship between variables, the explanatory variables are added in turn, and the changes of each explanatory variable coefficient in different models' values and significance levels are investigated. If there is little or no change, it is considered that the explanatory variable has a steady influence on the cognition and consumption intention of destination tourists.  Figure 6 shows the evaluation results of tourists' tourism.

It can be seen that tourists pay more attention to the bad environment, the quality of service, and the content of tourism activities when spending in tourist destinations. This paper examines the validity analysis of the scale by evaluating its discrimination validity and aggregation validity, among which structural validity is one of the most important validity indicators. Descriptive statistics of homesickness scale for tourists before and after the tour are shown in Table 5.

It can be seen that the “homesickness” emotion of tourists before traveling is mainly positive emotion. Most tourists will have feelings of excitement, pleasure, comfort, love, etc. before starting the trip of rural tourism, which shows that most tourists have positive feelings before rural tourism. Most tourists still have positive feelings after their trip to the countryside, but compared with before the trip, their positive feelings have decreased and negative feelings have slightly increased. The impact of homesickness emotional experience on tourists' consumption intention is shown in Figure 7.

RETRACTED

The research can draw the following conclusions:

The social, cultural, and economic environment in which consumers live is a changing environment, so people's values, aesthetic tendency, code of conduct, and consumption level will also change. However, the negative homesickness of rural tourists before the tour has a significant negative impact on their attribute perception and consumption intention and a significant positive impact on their negative homesickness after the tour, but not on their emotional perception. Rural tourists' perception of the attributes of tourist destinations has a significant positive impact on the positive homesickness after consumption and tourists' satisfaction, but it has no significant impact on the negative homesickness after travel. After the purchase of tourism consumption, tourists will have a general evaluation of the overall image of tourism products and tourism satisfaction under the influence of homesickness emotional experience. These evaluations will enrich the tourists' consumption experience, which will affect the tourists' decision-making in the next period. It is suggested that relevant departments and staff should pay attention to the excavation of “homesickness emotion” and arouse the emotional resonance of tourists; focus on creating rural tourism attractions; optimize the rural tourism experience of tourists.

## 5. Conclusions

The hidden behavior of big data is gradually emerging from the water as a result of its widespread application. Big data analysis allows for the segmentation of consumer behavior and the creation of customized marketing campaigns and services for each consumer group. This research studies the cognition of homesickness emotional experience to rural tourist sites and consumption willingness based on big data technology. This research examines the behavior traits of consumers' purchase intentions from the perspective of a “big data” environment, and as a result, it constructs the appropriate consumption behavior model of rural visitors. The impact of homesickness on the cognition and consumption intention of tourist locations is also investigated using qualitative analysis, logistic empirical analysis, and questionnaire survey. The research shows that the MSE of this algorithm is about 4.16, and the RMSE of this algorithm is about 0.508. In addition, rural tourists' negative homesickness before the tour has a significant negative impact on their attribute perception and consumption intention, a significant positive impact on their negative homesickness after the tour, and no significant impact on their emotional perception. Rural tourists' perception of the attributes of tourist destinations has a significant positive impact on the positive homesickness after consumption and tourists' satisfaction, but it has no significant impact on the negative homesickness after travel. After the purchase of tourism consumption, tourists will have a general evaluation of the overall image of tourism products and tourism satisfaction under the influence of homesickness emotional experience. These evaluations will enrich the tourists' consumption experience, which will affect the tourists' decision-making in the next period. Through the construction of consumer behavior model of rural tourism, this paper can enrich the research content of rural tourism in theory and help to understand the market rules of rural tourism scientifically. In practice, it is of great guiding significance for rural tourism enterprises to carry out project development, scientifically locate the market, find the target market, and choose marketing channels.

RETRACTED

## Figures and Tables

**Figure 1:** Relationship between attitude and tourism decision-making process.

**Figure 2:** The best point of tourist distance.

**Figure 3:** MSE results of different algorithms.

**Figure 4:** RMSE results of different algorithms.

**Figure 5:** Accuracy test results.

**Figure 6:** Evaluation results of tourists' tourism.

**Figure 7:** The impact of homesickness emotional experience on tourists' consumption intention.

**Table 1:** Rural tourists' homesickness scale.

Variable	Index
Travel to the front of homesickness (PPN)	PPN1: excited
	PPN2: pleasant
	PPN3: comfortable
	PPN4: favorite

Travel before negative homesickness (PNN)	PNN1: depressed
	PNN2: sad
	PNN3: disgusting
	PNN4: depressed

Travel back to the front homesickness (PN)	PPN1: excited
	PPN2: pleasant
	PPN3: comfortable
	PPN4: favorite

Negative homesickness after traveling (NN)	NN1: angry
	NN2: sad
	NN3: irritable
	NN4: regretful

**Table 2:** Survey of the sample of the investigator.

	Project and content	Total number of people
Rural tourism experience	0 times	19
	2 times	60
	3 times or more	52

Tourist source land	Tourists from other places	36
	Local resident	150

Gender	Man	88
	Woman	90

Monthly income	Less than 2000 yuan	48
	2001-4000 yuan	75
	4001-6000 yuan	42
	More than 6001 yuan	20

Age	Under 18 years old	5
	18-40 years old	86
	41-65 years old	98
	Over 66 years old	2

Degree of education	Junior high school and below	15
	Senior high school	50
	University	106
	Graduate student or above	40

Occupation	Staff of administrative organs, enterprises, and institutions	78
	Self-employed households	20
	Student	26
	Other	63

**Table 3:** Reliability test results of survey data.

Variable	Number of entry	Cronbach's alpha coefficient
Nostalgia emotion	6	0.778
Attitude of tourists	4	0.879
Willingness to consume	4	0.821

RETRACTED

**Table 4:** Descriptive statistics of tourist perception scale.

Variable	Topic item	Standard deviation
Attribute perception	AE1: beautiful scenery	0.711
	AE2: the regional characteristics of the destination are outstanding	0.729
	AE3: complete infrastructure	0.698
	AE4: there are many interactions with local residents	0. 781
	AE5: the service attitude and quality are very high	0.772

Emotional perception	EE1: appreciate the unique beauty	0.839
	EE2: feel the traditional culture and history of the countryside	0.768
	EE3: it's a wonderful memory	0.979

**(a):** 

Variable	Topic item	Standard deviation
Travel to the front of homesickness (PPN)	PPN1: excited	0.782
	PPN2: pleasant	0.721
	PPN3: comfortable	0.719
	PPN4: favorite	0.891

Travel before negative homesickness (PNN)	PNN1: depressed	1.006
	PNN2: sad	0.981
	PNN3: disgusting	0.919
	PNN4: depressed	0.948

**(b):** 

Potential variable	Topic item	Standard deviation
Travel back to the front homesickness (PN)	PPN1: excited	0.809
	PPN2: pleasant	0.812
	PPN3: comfortable	0.826
	PPN4: favorite	0.877

Negative homesickness after traveling (NN)	NN1: angry	1.136
	NN2: sad	1.009
	NN3: irritable	1.068
	NN4: regretful	1.075

## Data Availability

The data used to support the findings of this study are available from the corresponding author upon request.
